RETRACTED

# The Influence of Culture and Art Management on the Healthy Development of Cultural Economy Industry under the Background of Sustainable Ecological Environment

**DOI:** 10.1155/2022/3859292

**Published:** 2022-09-13

**Authors:** Jingyi Xu, Jianxin Wang, Qingyang Liu, Ziyan Xie, Lee Seo Jae, Avera Fiaidhi, Elvan Marcos

**Affiliations:** ^1^Department of Business, Gachon University, Seongnam-Si 13120, Gyeonggi Province, Republic of Korea; ^2^Information Science and Engineering, Chongqing Jiaotong University, 400074 Chongqing, China; ^3^Hubei University of Technology, Wuhan, China 430068; ^4^Changsha University, Changsha, China 410022; ^5^Kookmin University, Seoul, Republic of Korea; ^6^Lakehead, Lakehead University, Canada; ^7^Iloilo Science and Technology University, Iloilo, Philippines

## Abstract

In the context of sustainable ecological environment, strengthening the scientific management of cultural industry can promote the rapid development of China's cultural industry and further promote the construction of spiritual civilization in China. Starting from culture and art management, this study expounds its position in the development of cultural economy industry and its impact on the development of cultural economy. Through two different methods of culture and art management and conventional management, this paper discusses the social and economic market benefit value, the demand for the healthy development of industry, and the impact of innovative cultural industry resources on the development of cultural industry. It can be concluded that culture and art management plays a certain role in promoting the healthy development of cultural economy industry; we should constantly sum up experience in the actual process of cultural industry management, find and solve problems in time, and gradually form a set of scientific and complete cultural and art management mode, which can realize the transformation of cultural and art industry faster and better promote the sustainable development of cultural economy and industry.

## 1. Introduction

With the continuous improvement of the national economic level, China's cultural and economic industry has entered a period of prosperity and development. But there are also many problems, such as the instability of the industrial system. Various problems have hindered the further development of the cultural and economic industry, so we must pay attention to the role of cultural and artistic management, and let cultural and artistic management maintain and promote the healthy development of the cultural and economic industry. Culture and art management is not the product of modern society. Culture and art management has existed in the pre-Qin period of our country. However, the requirements for culture and art management are different in each era. Xialu [1] said that in the new era, the development situation of China's culture and art presents new characteristics, and the management of culture and art must change accordingly. The management of culture and art should pay attention to the cultivation of management talents, give full play to the role of management talents, and attach great importance to the improvement of culture and art management level, so as to promote the development of China's cultural industry and finally realize the development of culture and art management.

RETRACTED

Lei [2] said that the important concept of contemporary Chinese culture and art management is to promote the all-round development of people and society. In the current context of sustainable ecological environment, in order to enable the cultural and economic industry to develop healthily and stably, appropriate changes should be made in the management of culture and art, so as to better guide the cultural and economic industry. Jing [3] believes that the culture and art industry is a kind of consciousness oriented behavior, which guides people's behavior orientation and has a great impact on the public. Some western capitalist countries have realized this problem and formed an ideological development system suitable for capitalist society. China's culture and art management should also draw on Western experience, give play to the driving and guiding value of culture, and provide favorable conditions for the construction of a benign cultural industry development system. Jing [4] and others said that culture and art management can strengthen the role of the main body of cultural industry management (government), ensure the mainstream cultural awareness of the communication content, and create a healthy space for the development of culture and art. At the same time, culture and art management can enhance the market vitality of the cultural industry, improve the activity of the main body of the cultural industry market, and help to further strengthen and optimize the culture and art market. Wei [5] said that contemporary Chinese society is in an important historical stage of building cultural self-confidence and cultivating core socialist values. Literary and artistic creation is the pillar force of cultural construction. Literary and artistic creation needs an atmosphere and environment in which a hundred flowers bloom and a hundred schools of thought contend; otherwise, its vitality and innovation will be affected. Therefore, the administrative management of culture and art by government departments should not be too much and too detailed, but should rely on the aesthetic governance and cultural governance functions of art criticism.

RETRACTED

The cultural industry is an important part of China's economic industry. According to the accounting, the total added value of the national cultural and related industries in 2020 was 4494.5 billion yuan, an increase of 1.3% over the previous year, accounting for 4.43% of the gross domestic product (GDP). While it has an impact on the development of the national economy, it also plays an important guiding role in the cultural literacy of the people. In the context of sustainable ecological environment, the purpose of culture and art management is to continuously improve the innovation and development level of the cultural industry and promote the healthy and orderly development of the cultural economic industry. Xin [6] said that when developing the cultural industry, we should pay attention to the management of culture and art. Only in this way can we effectively guide and manage the development of the cultural industry and ensure that the cultural industry can actively respond to the development of the times and win the favor of the masses [6]. Zeqian [7] said that the important role of the management of culture and art in the cultural industry is concentrated in the following aspects: There are essential differences between culture and art management and other types of production management. The implementation of management for culture and art is mainly to implement special management and planning for cultural and art works, and visually present cultural and art works to the public, so as to promote the continuous improvement of people's cultural literacy and aesthetic literacy [7]. Rikui [8] believes that at present, if we want to improve the influence and dissemination of China's cultural industry, we must scientifically and effectively carry out cultural and art management to provide strong support and guarantee for the prosperity and development of the cultural industry. Qianhong [9] pointed out that China's cultural and economic industry has developed rapidly, but it has not formed a specific market system, and its development level is low, which cannot effectively meet people's spiritual needs. There will be some problems in the specific development process, so it is necessary to further strengthen cultural and art management. Tianyue [10] expressed the same view. He believes that we should strengthen the management of culture and art, improve the quality of culture and art products while improving economic benefits, and take various measures to improve the management level of culture and art on the basis of respecting the reality of the development of China's cultural industry. Xiaoying [11] and others believe that we must recognize the importance of culture and art management for realizing the development strategy of cultural economy industry. Culture and art management can change the focus of the development of cultural economy industry, purify its development environment, break the shackles of costs on its management mechanism and scientific research work, and truly promote the standardized and comprehensive development of cultural economy industry [11].

RETRACTED

This paper mainly focuses on the impact of cultural and art management on the healthy development of cultural and economic industries under the background of sustainable ecological environment, hoping to provide reference value for the field of cultural and economic industries through this research and contribute to the stable and harmonious development of cultural and economic industries in our society.

## 2. Overview of Culture and Art Management

Culture and art management is a purposeful and all-round management behavior for culture and art activities. In short, it is to manage culture and art in all aspects, so as to achieve better artistic effects and create more profitable products for the cultural and economic industry. At the same time, cultural and artistic products have a great impact on people's spirit. Excellent cultural and artistic products can enrich people's spiritual world and improve cultural and aesthetic literacy at the same time. Therefore, strengthening the management of cultural industry is of great significance to the long-term development of cultural industry.

Industrial products can attract consumers by reducing prices, but cultural products cannot. High-quality cultural products can meet people's cultural needs and have a positive impact on people. Low-quality cultural products will have a negative impact on people, leading to depression, degeneration, or violence. If the cultural market is full of too many low-quality products with distorted values, it will hinder the healthy development of the cultural economic market and harm the society. At present, the cultural and economic industry is developing rapidly. In order to earn immediate benefits, many people deliberately manufacture low-quality and eye-catching cultural products, disrupting the normal operation of the cultural and economic industry. Therefore, it is necessary to carry out scientific management of the cultural and economic industry. It can be said that culture and art management is an important productive force for the development of cultural industry and a production factor to create economic benefits. Culture and art management is not only the management of cultural activities, but also the management of cultural ideology.

RETRACTED

In culture and art management, culture and art managers play an important guiding role. Under the impact of current multiculturalism, how China's cultural and economic industry can go better, further and more in line with the core socialist values, is a problem that cultural and art managers need to think about and solve. At present, China does not pay enough attention to the management of the cultural and economic industry, and does not solve the problems existing in the cultural industry in time. At the same time, there are not enough professional cultural management talents. Some of the existing cultural managers have insufficient experience, do not correctly recognize the influence of the cultural industry, and have weak awareness of innovation and responsibility. Therefore, the development of cultural and art management in China lags behind.

## 3. The Position of Culture and Art Management in the Development of Cultural Economy Industry

In the context of sustainable ecological environment, culture and art management should closely follow the pace of cultural development, and at the same time, we should clearly recognize the important position of culture and art management in the development of cultural economic industry. In the process of the development of the cultural industry, it is very likely to deviate from the normal development track. Therefore, the guiding role of management orientation is highlighted. The improvement of the comprehensive ability of managers meets the cultural needs of consumers at the spiritual level, actively carries out the pursuit of healthy spiritual culture, abandons the previous bad culture, and better implements the rectification of the social environment. The management of culture and art does not only focus on the art itself. It also includes other management elements.

The upsurge of cultural consumption has stimulated consumers' enthusiasm for cultural consumption, expanded the demand of the cultural market, and improved consumers' level of cultural consumption, and consumption has stimulated economic growth, which has a positive role in promoting cultural and creation. In today's society, the cultural industry, as a country's soft power, has increasingly highlighted the economic function of culture, which affects the development of economic society in the characteristics of strong permeability and durability. Pay attention to the scientific nature of management. Its management is an important productive force in industrial development, a thrust to improve the level and create fine products in the development of cultural industry, and a production factor that produces economic benefits. The role of culture in promoting, guiding, and supporting economic development has become more and more obvious. In order to develop cultural and artistic works in art management to meet the spiritual needs of consumers, cultural and artistic management should develop in the direction of strengthening the foundation and emphasizing humanities, so as to promote the long-term development of art management.

RETRACTED

Different from other industries, the cultural industry has special spiritual and cultural social attributes. Its special attributes determine the primary position of social benefits. The cultural industry should maintain the vitality of healthy development. The cultural industry, which carries social and educational functions, meets the needs of consumers for a better life to the greatest extent, and clearly guides the sustainable and healthy development of the cultural and economic industry, so as to enhance its initiative of sustainable development.

## 4. Influence of Culture and Art Management on the Development of Cultural Economy

Culture and art management has a far-reaching impact on the sustainable development of culture and economy. Culture and art management is the standardized and orderly management of the actual needs of the development of China's culture and art industry. Only in this way can we increase cultural competitiveness, form a standardized operation mechanism, provide favorable conditions for promoting the development of culture and economy, strengthen management, and give play to the positive guiding influence of management. Give full play to the driving and guiding value of culture, and build a virtuous cycle of industrial development system. Cultural and economic industries can not only create higher economic benefits, but also promote the benign development of society, especially the culture with positive guiding significance.

In this study, culture and art management is used for the application and in-depth excavation of cultural resources to improve its management level. Product research and development and management itself play an important role in promoting creation. Therefore, the development of scientific and feasible management measures can play an important role in getting twice the result with half the effort and creating more and more popular cultural and art works. Today, management has been characterized by profitable development. Considering the particularity of culture and art management, it is necessary to strengthen management simulation to prevent cultural distortion. It can indirectly enhance the influence of China's cultural industry and actively promote the cultural industry to go wider. As a special cultural form and special economic form, the cultural industry has affected the people's grasp of the essence of the cultural industry. Under the guidance of norms, we should strive to write a new chapter of cultural development and prosperity.

RETRACTED

Culture and art management plays a key role in the development of cultural industry. Formulate reasonable management countermeasures, push the cultural industry to a new level of development, promote a clear operation direction in the guiding trend, move in a good direction, and comprehensively improve the cultural soft power, cultural competitiveness, and cultural sustainable development ability. Now, according to the culture and art management oriented trend from 2012 to 2021, the obtained data are made into Figure 1 as follows.

As shown in Figure 1, it can be seen that the concept of culture and art management has been paid more and more attention. With the passage of years, the development direction of the cultural economy industry has become clearer and clearer. Under the background of sustainable ecological environment, culture and art management has played a key role in the development of the cultural industry.

## 5. Simulation Verification

### 5.1. Analysis of Industrial Development Efficiency under Different Management

Cultural industry is an important part of China's economic development and is of great significance to China's economic development. Constantly strengthen the management of cultural products, promote the sustainable development of cultural and economic industries, and maximize the market economic benefits of cultural and artistic products while doing a good job in cultural and artistic management. Conventional management methods do not pay enough attention to the development of economic industries, which is not conducive to the development of cultural industries. Now, the effectiveness of two different management methods on the healthy development of the industry is analyzed, and the data obtained are made into Table 1 as follows.

In Table 1, the data analysis of the development efficiency of culture and art management shows that its management mode has broken the unbalanced state of resource allocation. Taking into account the preferences and aesthetic views of consumers, we should strengthen efforts to develop innovative art products, create them in combination with the characteristics of practicality and artistry, expand its market influence, increase the value of market benefits, and promote the virtuous development cycle of culture.

The visual analysis of the above data results is made into Figure 2 as follows.

RETRACTED

As shown in Figure 2, the effectiveness analysis of applied culture and art management for the healthy development of the industry is significantly higher than that of conventional management. From the analysis results, it is obvious that the cultural and economic industries can be better integrated with the development of the times and lay a solid foundation for the healthy development of cultural and economic industries.

### 5.2. Comparison of Industrial Healthy Development Needs under Different Management

In order to improve the quality of cultural and art management and comprehensively improve its management effect, we need to improve the comprehensive ability of cultural managers. If we want to have a better development of cultural products, we must ensure that cultural and art management has high-quality support, strengthen cultural and art management mechanism, and promote the sustainable development and progress of cultural and art management. The research and development of cultural and art products will promote the better development of cultural and economic industry. In the process of paying attention to the development of cultural and economic industries, we must do a good job in the management of culture and art to fundamentally provide the foundation for the cultural industry. Now, we compare the needs of two different management methods for the healthy development of the industry and make the obtained data into Table 2 as follows.

In Table 2, the demand for the healthy development of the cultural and economic industry in the management and operation mechanism, the comprehensive ability of managers, and the research and development of art products is clear, and the healthy development demand of the industry under the conventional management mode are significantly lower than the management mode used in this study. Bivariate *t*-test was performed on the corresponding data in pairs, and there was a test result of *t* < 10.000 and *p* < 0.05, which was statistically significant between the data.

The visual analysis of the above data results is made into Figure 3 as follows.

As shown in Figure 3, culture and art management is significantly higher than conventional management in all aspects of the healthy development needs of the industry. It can be considered that cultural and art management will gradually improve the impact of the cultural industry. Implementing a reasonable management mechanism in the process of management and paying attention to the comprehensive ability of personnel can provide favorable conditions for the follow-up research and development of cultural products.

### 5.3. Benefit Analysis of Industrial Development under Different Management

The development of cultural and economic industries has been raised to a strategic height, creating an atmosphere that attaches importance to the development of cultural industries, and vigorously promoting the development of cultural industries. The management of culture and art improves the quality of cultural and artistic products while improving social and economic benefits. In the previous conventional management, the cultural market cannot perfectly adapt to the situation of cultural and artistic development, and cultural products also lack artistry. It is not in line with public aesthetics, which seriously hinders and restricts the development of the cultural industry. This study adopts the cultural and artistic management method to innovate cultural and artistic products and carries out reasonable management and subsequent arrangements for the development of the cultural industry to further promote the green and sustainable development of the industry. Now, the effects of two different management methods on the benefits of industrial sustainable development are compared, and the data obtained are made into Table 3 as follows.

RETRACTED

In Table 3, the cultural and art management method is adopted to understand the needs of consumers for the market and innovate and enrich the diversity of cultural and art industry resources. According to the current cultural development trend, it breaks the shackles of the traditional cultural industry, expands its market development influence, promotes the comprehensive and sustainable development of the cultural industry, and greatly improves the social and economic benefits.

The visual analysis of the above data results is made into Figure 4 as follows.

As shown in Figure 4, it can be clearly seen that the industrial development benefits of the two groups of different management methods have widened the gap in innovative cultural industry resources, cultural industry development influence, and social and economic benefits, indirectly indicating that cultural and art management can effectively promote social and economic benefits, and cultural industry has become an important way of economic growth in economic development.

## 6. Summary

In recent years, in order to meet the needs of social development and solve the problem of the shortage of professionals in the cultural industry, China has set up a new management discipline—culture and art management, which is based on literary theory and aims at the development needs of social and cultural production, and has cultivated a number of senior comprehensive talents. Culture and art management plays an important role in the healthy development of cultural economic industry. In the current context of sustainable ecological environment, we must pay attention to the cultural and economic industry with green environmental protection and high-added value. Therefore, it is essential to establish a scientific culture and art management system and establish a scientific culture and art management system. Xingyu [12] said that culture and art management should face the future. Its productivity is embodied in intelligent technology, its means of production is embodied in Chinese culture, and its production relations are embodied in building an international vision. This is an important goal of culture and art management thinking [12]. Attaching importance to culture and art management is an important measure to develop the cultural and economic industry. We should follow the development path of China's socialist cultural characteristics, strengthen innovative thinking, and explore a culture and art management path that suits China's national conditions, so as to further accelerate the development of the cultural industry, provide impetus for the cultural and economic industry, and promote the long-term development of the cultural and economic industry.

RETRACTED

## Figures and Tables

**Figure 1:** Trend chart of culture and art management in different years.

**Figure 2:** Visualization of industrial development efficiency under different management (%).

**Figure 3:** Visualization of industrial healthy development demand under different management (%).

**Figure 4:** Visualization of the impact of industrial sustainable development benefits under different management (%).

**Table 1:** Analysis of industrial development efficiency under different management (%).

Group	Market benefit value	Resource allocation and distribution	Cultural development cycle
Culture and art management	85.56	84.64	85.29
General management	67.73	63.48	64.53

**Table 2:** Comparison of industrial healthy development demand under different management (%).

Group	Management and operation mechanism	Comprehensive ability of cultural management personnel	Research and development of cultural and artistic products
Culture and art management	80.32	83.64	85.45
General management	65.78	64.72	64.38

**Table 3:** Impact analysis of industrial sustainable development benefits under different management (%).

Group	Innovative cultural industry resources	Cultural industry development influence	Social and economic benefits
Culture and art management	90.62	89.32	92.38
General management	70.45	68.45	71.33

## Data Availability

The data underlying the results presented in the study are available within the manuscript.
